The article "BJBN： BERT-JOIN-BiLSTM Networks for Medical Auxiliary Diagnostic" was retracted in 2023. Reasons: signs of a paper mill; suspected computer-generated content; unreliable results or conclusions; concerns about the data.

# BJBN： BERT-JOIN-BiLSTM Networks for Medical Auxiliary Diagnostic

**DOI:** 10.1155/2022/3496810

**Published:** 2022-01-11

**Authors:** Chuanjie Xu, Feng Yuan, Shouqiang Chen

**Affiliations:** ^1^Shandong Provincial Key Laboratory for Novel Distributed Computer Software Technology, Jinan, China; ^2^School of Information Engineering, Shandong Management University, Jinan 250357, China; ^3^Center of Hear of the Second Afﬁliated Hospital of Shandong University of Traditional Chinese Medicine, Jinan 250001, China

## Abstract

This study proposed a medicine auxiliary diagnosis model based on neural network. The model combines a bidirectional long short-term memory（Bi-LSTM）network and bidirectional encoder representations from transformers (BERT), which can well complete the extraction of local features of Chinese medicine texts. BERT can learn the global information of the text, so use BERT to get the global representation of medical text and then use Bi-LSTM to extract local features. We conducted a large number of comparative experiments on datasets. The results show that the proposed model has significant advantages over the state-of-the-art baseline model. The accuracy of the proposed model is 0.75.

## 1. Introduction

At present, medical diagnosis is mostly based on the information obtained from the diagnosis of equipment and instruments, combined with the medical knowledge of physicians and years of accumulated experience for diagnosis. However, in the process of diagnosis, the subjectivity of the doctor may cause misdiagnosis in the process of diagnostic reasoning, which reduces the accuracy of manual diagnosis and weakens the confidence of patients in clinical practice [1, 2].

To solve this problem, researchers have proposed auxiliary models for clinical diagnosis and treatment [3, 4]. Specifically, the goal of the model is to predict the final diagnosis based on TCM symptoms as the input; for example, when we input relief of chest tightness but persistent tiredness and sluggishness, the model predicts a diagnosis of chest paralysis. Such a model can help practitioners use medical knowledge to more effectively solve various medical problems and make clinical diagnosis and decision-making faster, avoid omissions, and prevent the loss of relevant information, to find more solutions to intractable diseases [5, 6]. In view of this, this paper studies a new medical-assisted diagnosis model. Due to differences in individual levels of experience and research purposes, the conclusions reached from models can be relatively subjective as well as both time-consuming and difficult to implement in the clinic. Therefore, it is necessary to introduce new technologies and methods to quickly ascertain the doctors' research goals and clinical experience from massive amounts of medical data. In recent years, with the development of artificial intelligence, especially deep learning, more and more neural network technologies are applied to intelligent diagnosis. For example, modelling using neural networks and random forests shows high accuracy in clinical diagnosis with multicategory classification [7–9]. Although these models circumvent some of the problems of traditional methods, they still have great deficiencies in the acquisition of medical text information. So, the model's understanding of medical texts must be strengthened.

In this paper, a medical-assisted diagnosis model based on Bi-LSTM network and BERT was proposed. Bi-LSTM can better capture the information of the sentence and improving the classification performance of the sequence [10, 11]. BERT can generate a deeper two-way language representation; the word vector can contain more contextual information [12, 13]. The model can complete five categories of classification tasks and can effectively enhance the understanding of the local features of TCM texts, thereby improving the accuracy of the model for predicting diseases.

The main contributions of our work can be summarized as follows:

1. A model based on Bi-LSTM and BERT was proposed for medical-assisted diagnosis
2. Incorporating global information into the extraction of local features can obtain more local features of the text
3. The proposed model can also be fine-tuned to apply it to other professional fields

## 2. Related Work

At present, there are few studies on auxiliary diagnosis systems for clinical texts and those that do focus on English clinical texts and feature engineering; very little work exists on Chinese clinical texts and deep learning models. The method used for the auxiliary diagnosis model at the beginning is the comprehensive analysis method. Mi et al. [14] combined different data mining technologies and proposed a personal understanding and statistical analysis method to explore the dialectics and treatment rules of TCM-based disease treatment and obtain valuable information from them. With the development of machine learning, especially deep learning, many researchers apply it to auxiliary diagnosis. Chen et al. [15] applied support vector machines and decision trees to the classification of breast cancer texts and achieved good results. Ekong et al. [16] used the fuzzy clustering method to detect liver function patients. Xu et al. [17] designed and implemented a medical information text classification system based on a KNN. In addition, the three main deep learning models for auxiliary diagnosis are convolutional neural networks (CNNs) [18], recurrent neural networks (RNNs) [19], and FastText [20]. Zhang et al. [21] proposed an auxiliary diagnosis method based on a convolutional neural network. This model can diagnose the patient's condition through the wrist pulse. Kale et al. [22] applied a modern LSTM method to large datasets of multiple clinical time series for the first time and achieved certain results. Hu et al. [23] proposed a model that can be used to assist in diagnosis by calculating the Yin and Yang dialectic based on FastText. The input to these models can be words or characters. Although these models have achieved certain results, their understanding of the texts remains insufficient. Our proposed auxiliary diagnosis model can effectively solve this problem.

## 3. Model

The proposed model is shown in Figure 1. In this model, the bidirectional encoder representations from transformers (BERT) first obtains the global representation of the input text, then integrates the global information into the local information when extracting the local information, and finally performs the feature of the local information integrated into the global information. Extract and output the final prediction results.

### 3.1. BERT

First, we use BERT to get global information; the model architecture of BERT is based on the original transformer model. The input representation is a concatenation of WordPiece embeddings, positional embedding, and the segment embedding. Specifically, for single sentence classiﬁcation, the segment embedding has no discrimination. Let *W_t_* be the vector representation of the *t*th word in a sentence of length *n*; then, use BERT to encode to get *h_t_*:

(1) $$\begin{array}{c} h_{t}=BERT\left(w_{t}\right). \end{array}$$

The BERT model is pretrained on unlabeled large-scale texts through two strategies, namely, shielding language modelling and next sentence prediction. The pretrained BERT token embedding provides a powerful context-sensitive utterance representation, which can be used in various target models, such as TextCNN and Bi-LSTM. Many natural language processing (NLP) tasks benefit from the use of BERT to achieve state-of-the-art performance and reduce training time. The transformer structure of the component in BERT is shown in Figure 2.

### 3.2. Bi-LSTM

After obtaining the global information, we use the bidirectional recurrent neural network to extract the local features integrated into the global information, and the LSTM network, which includes a set of memory cells, is able to learn long-term dependencies. The structure of a single memory cell is presented in Figure 3. The LSTM network transmits the input information in two ways, as an output (or hidden) vector (denoted by h) and as a state vector (denoted by c), which are combined using three gates that are explicitly designed to store and propagate long-term dependencies.

Gate *i* is called the input gate. The value of its output will be updated in the state vector. The gate *f* is called the “forgotten gate,” which can determine which information in the previous state can be discarded. The storage unit uses the output of these two gates to create a new state vector. Finally, gate *o*, called the output gate, generates the final output vector of the memory cell. H represents the output of the current unit. The following equations are used in each memory cell to generate the output vector and state vector of the torque:

(2) $$\begin{array}{c} i_{t}=\delta \left(w_{xi}\cdot x_{t}+w_{hi}\cdot h_{t-1}+w_{ci}\cdot c_{t-1}+b_{i}\right),\\ f_{t}=\delta \left(w_{xf}\cdot x_{t}+w_{hf}\cdot h_{t-1}+w_{cf}\cdot c_{t-1}+b_{f}\right),\\ c_{t}=f_{t}\cdot c_{t-1}+i_{t}\cdot \text{tan}h\left(w_{xc}\cdot x_{t}+w_{hc}\cdot h_{t-1}+b_{c}\right),\\ o_{t}=\delta \left(w_{xo}\cdot x_{t}+w_{ho}\cdot h_{t-1}+w_{co}\cdot c_{t}+b_{o}\right),\\ h_{t}=o_{t}\cdot \text{tan}h\left(c_{t}\right). \end{array}$$

After inputting all sentences into BERT, all vector representations of the current text can be obtained:

(3) $$\begin{array}{c} H=\left[h_{1};h_{2};\ldots h_{n}\right]. \end{array}$$

Pass the obtained text vector through the average pooling layer to obtain the final global representation *g*:

(4) $$\begin{array}{c} g=\text{Average}\left(H\right). \end{array}$$

After obtaining *g*_, blend it into the middle of the local sequence and then use the recurrent neural network to extract its features. After extraction by the convolutional neural network, *L* is obtained:

(5) $$\begin{array}{c} L=\text{LSTM}\left(x_{t-1},g,x_{t}\right). \end{array}$$

After obtaining *L* through the recurrent neural network, pass it through the softmax layer to obtain the final prediction result PL:

(6) $$\begin{array}{c} \text{PL}=\text{softmax}\left(L\right). \end{array}$$

## 4. Experiment

Experimental results show that our model achieves state-of-the-art performance. All experiments were performed on an Nvidia GTX 1080 and RTX 2080Ti GPU.

### 4.1. Data

We used 20,000 TCM medical records collected from the outpatient clinic of the Second Affiliated Hospital of Shandong University of Traditional Chinese Medicine from 2015–2019 as the dataset. For those data that do not meet the writing standards of Chinese medicine and duplicate data, we use manual methods to remove them. Of the 20,000 records obtained, 2333 can be used for this experiment. One of the data samples is as follows: the main cause is suffocation, and patient's legs were swollen for two consecutive months. The patient was diagnosed as coronary heart disease and myocardial infarction due to chest pain and sweating 7 years ago. Medication was taken; CABG surgery was performed in the same year, and medication was persisted thereafter. In the past 3 years, chest tightness during activity occurred again, and nitroglycerin can be relieved quickly. In the past 1 year, shortness of breath and fatigue were caused by exertion, and it was easy to catch a cold. In the past 2 months, edema of both lower extremities occurred. The patient has symptoms such as cough, sputum, abdominal distension, anorexia, nausea, and cold. The complexion is yellow and white, the tongue is pale and dark with ecchymosis and tooth marks, and the pulse is heavy. These data are associated with 5 disease categories (chest paralysis, dysphoria, dizziness, palpitations, and thirst).  Figure 4 shows the percentage of various diseases.  Table 1 shows the specific number of each disease. The training set contains 1866 records, and the test set contains 467 records. The average number of characters in each record is 316. To ensure proper experimental results, we manually divided the dataset to create the training and test data. The ratio of the incidence of each disease in the training set to that of the test set is 4 : 1.

### 4.2. Detailed Description of the Experiment

In this study, the natural language toolkit (NLTK) is used in the preprocessing stage to process each question and its corresponding answer in the dataset. The processing includes case conversion, stemming reduction, and stop-word removal. The GloVe model proposed by Pennington et al. [24] was trained to obtain 300-dimensional initial word vectors, while the word vectors of words not in the dictionary were initialized to 300-dimensional zero vectors. Adam is used as the optimizer in this paper, with a first momentum coefficient of 0.9, a second momentum coefficient of 0.999, adaptive learning rates of [1 × 10^−9^, 4 × 10^−5^, 1 × 10^−7^], L2 parameters of [1 × 10^−6^, 4 × 10^−7^, 1 × 10^−7^], and batch sizes of [64,128,256]. We select the best parameters with the training set and then evaluate the final performance with the test dataset.

### 4.3. Experimental Results and Analysis

To evaluate the performance of the model proposed in this article, three indicators are used: F1-score, accuracy (Acc), and mean average of precision (MAP). We also use these indicators to compare the results of the proposed model with seven pre-existing classification models. These comparisons are shown in Table 2 in which (1), (2), (3), (4), (5), (6), and (7) correspond to [22, 23, 25–29], respectively, and (8) is the proposed method (baseline).

From the results of Table 2, we can draw the following conclusions:

1. The FastText model, based on *n*-grams, performs better than the TextCNN and TextRNN models in the three evaluation indexes (MAP, F1-score, and Acc) mainly because there are a large number of medical nouns in the experimental datasets used in this article, which are utilized by the *n*-grams feature, resulting in a better model performance. These results also prove that it is necessary to train the word vectors in special fields (Row1 vs. Row2 and Row3).
2. The TextRCNN method is superior to the TextCNN, TextRNN, and FastText models according to the three indicators used in this experiment. The main reason for this is that TextRCNN combines the advantages of the TextCNN and TextRNN models and makes them complementary. This result also proves that although the *n*-grams feature has an important role in the medical diagnostic process; as the architecture of the deep learning network model becomes more complicated, the effect of the *n*-grams feature will result in a worse performance than the deep learning model, which is why the deep learning model shines in various natural language processing tasks (Row4 vs. Row1, Row2, and Row3).
3. Compared with those for the deep pyramid convolutional neural network (DPCNN) method, the results obtained for the previous four methods are poor. This is because the DPCNN model is relatively complicated. At the same time, the datasets used in this article are mostly short text. Not all tasks using deep learning methods can achieve good results; we should choose the model that suits our needs for specific tasks in order to effectively obtain good results (Row5 vs. Row1, Row2, Row3, and Row4).
4. The TextRNN_Att method outperforms methods (1)–(5) in terms of the three evaluation indicators. This is because TextRNN_Att introduces the attention mechanism into TextRNN; this captures the displayed text sequence features and thus shows good results, further proving that the introduction of the attention mechanism is beneficial for medical auxiliary diagnostic tasks (Row6 vs. Row1, Row2, Row3, Row4, and Row5).
5. The transformer method only slightly outperforms the DPCNN method and is otherwise outperformed by several of the other models in terms of the three evaluation indicators. This is because most of the datasets used in this article are short text. Transformer is relatively complicated and therefore performs poorly when capturing short text features. These results further prove that the Transformer model is not suitable for medical auxiliary diagnostic tasks (Row7 vs. Row1, Row2, Row3, Row4, Row5, and Row6).
6. The medical-assisted diagnosis method proposed in this paper to enhance local feature extraction has higher MAP, F1, and Acc values than all the above models. It can be seen that the proposed model can effectively use global information to enhance the local information of medical text extraction ability, which also shows that the method proposed in this paper is an effective medical-assisted diagnosis method.

### 4.4. Parameter Sensitivity

In this section, we evaluate the impact of some parameters such as hidden state dimension of Bi-LSTMs on our dataset.

We investigate the impact of hidden state dimension of LSTMs with results shown in Figure 5. We can see that Acc of our model shows an upward trend when the dimension size is less than 300, especially achieving highest when the dimension size is exactly 300, which indicates that a large dimension size could contribute to model performance. However, when the dimension size is larger than 300, the accuracy of the model drops on both development sets and test sets possibly due to insufficient training data.

## 5. Conclusion

In this paper, the medical auxiliary diagnosis model is studied by using a real-world medical dataset, leading to the proposal of a new model to address the shortcomings of existing methods. The experimental results show that our proposed model has certain advantages over previous models in medical auxiliary diagnosis. The main results of this paper can be summarized in two points. (1) A model based on Bi-LSTM and BERT was proposed for medical-assisted diagnosis. (2) Our work of this paper can have an inspirational effect on research in related fields.

Our experimental results show that the proposed auxiliary diagnostic model can obtain better results than the previous classic model, achieving an accuracy of 75.69%, which is very competitive with recently published auxiliary diagnostic models.

## Figures and Tables

**Figure 1:** BJBN network model.

**Figure 2:** Transformer model structure.

**Figure 3:** The structure of a memory cell.

**Figure 4:** Percentage of the Chinese medical record datasets by symptom.

**Figure 5:** The influence of Bi-LSTM dimensions on experimental results.

**Table 1:** The corpus size of the dataset of Chinese medical records.

Data set	Symptom name	Number of medical records	Number of characters
TCM data	Chest pain	826	261016
	Dysphoria	453	143148
	Dizziness	360	113760
	Palpitations	349	100804
	Thirst	345	109020

**Table 2:** Experimental results of eight models with TCM data.

Model	Average acc	Average precision	Average recall	Average F1-score
FastText	0.6628	0.7520	0.5866	0.6592
TextCNN	0.6243	0.7362	0.5621	0.6375
TextRNN	0.6521	0.7456	0.5697	0.6459
TextRCNN	0.6957	0.7672	0.6238	0.6881
DPCNN	0.6139	0.6692	0.5873	0.6256
TextRNN_Att	0.7153	0.7749	0.6477	0.7056
Transformer	0.6285	0.6837	0.5891	0.6329
Our model	0.7512	0.8352	0.6818	0.7569

## Data Availability

The data used to support the findings of this study are available from the corresponding author upon request.
